# MCOLN1 Promotes Proliferation and Predicts Poor Survival of Patients with Pancreatic Ductal Adenocarcinoma

**DOI:** 10.1155/2019/9436047

**Published:** 2019-08-05

**Authors:** Zhan-Dong Hu, Jun Yan, Kai-Yue Cao, Zhi-Qi Yin, Wei-Wei Xin, Ming-Fang Zhang

**Affiliations:** Department of Pathology, Tianjin First Central Hospital, Number 24, Convalescent Road, Nankai District, Tianjin 300192, China

## Abstract

**Background:**

MCOLN1 (mucolipin subfamily, member 1) was first identified as an autophagic regulator, which was essential for efficient fusion of both autophagosomes and late endosomes with lysosomes. This study is aimed at investigating the role of MCOLN1 in the development of pancreatic ductal adenocarcinoma (PDAC).

**Methods:**

Immunohistochemistry (IHC) assay was conducted to evaluate the expression level of MCOLN1 in 82 human PDAC tumor tissues. Overall survival (OS) and recurrence-free survival (RFS) analysis was performed to assess the prognosis of patients. Colony formation and MTT assays [3-(4,5-dimethyl-2-thiazolyl)-2,5-diphenyl-2-H-tetrazolium bromide] were performed to measure the proliferation capacity of tumor cells. The expression level of related genes was measured by RT-PCR (reverse transcription polymerase chain reaction) and western blot assays. The animal model was used to examine the effects of indicated protein on tumorigenesis in vivo.

**Results:**

The results of IHC showed that a high level of MCOLN1 expression was associated with the poor clinical characteristics of PDAC patients. OS and RFS were significantly worse in patients with high MCOLN1 expression. Silencing of MCOLN1 dramatically blocked the proliferation of PDAC cells. Mechanism studies confirmed that knockdown of MCOLN1 decreased the expression of Ki67 and PCNA (proliferating cell nuclear antigen), two markers of cell proliferation. In vivo, MCOILN1 depletion reduced the formation and growth of tumors in mice.

**Conclusion:**

The high level of MCOLN1 expression was associated with poor clinical outcomes of PDAC patients. MCOLN1 ablation could inhibit PDAC proliferation of both in vitro and in vivo, which provide a new insight and novel therapeutic target for the treatment of PDAC.

## 1. Introduction

Pancreatic cancer is a type of common digestive system carcinoma with 56,770 newly diagnosed cases and 45,750 deaths estimated in USA 2019 and is predicted to become the second main cause of cancer-related deaths by 2030 [1, 2]. Among the types of pancreatic cancers, pancreatic ductal adenocarcinoma (PDAC) accounts for about 90% [3]. Despite the advances of combined treatment strategies and the improvement of techniques including surgery, chemotherapy, and immunotherapy, the prognosis of patients is still poor, with a 5-year survival rate of 6% [4]. Although various gene signatures and signaling pathways have been found to participate in tumor progression in recent years, the precise mechanism of PDAC progression is extraordinarily perplexed and heterogeneous and has not been completely understood [4–7].

MCOLN1 (mucolipin subfamily, member 1), also known as mucolipin-1 or TRPML1 (transient receptor potential cation channel, mucolipin subfamily, member 1), is the best-characterized member of the TRPML family since the mutations of this protein were associated with mucolipidosis type IV (MLIV), a devastating neurodegenerative disease [8, 9]. Primarily residing in the membranes of late endosomes and lysosomes, MCOLN1 is a Ca^2+^ channel that releases lysosomal Ca^2+^ and may regulate fusion/fission of vesicles through the endocytic pathway [10–13]. Specially, in 2019, MCOLN1 was reported as a promotor to regulate mTORC1 and purinergic signaling pathways in the development of triple-negative breast cancer [14]. In mammal cells, mouse macrophages with reduced expression of MCOLN1 show delayed transport of fluid-phased factors to lysosomes, impaired exit of LacCer from lysosomes, and reduced transport of major histocompatibility complex (MHC) II to the plasma membrane [15]. Besides, MCOLN1 was reported to protect against imidazole-induced cytotoxicity. Also, inhibition of MCOLN1 resulted in severe combined immunodeficiency diseases [16, 17]. However, the potential role of MCOLN1 in human carcinoma development has not been studied clearly.

Among the TRP family, mucolipins represented a distinct subfamily of endosome/lysosome Ca^2+^ channel proteins [18–25]. The TRPML channels were 6 transmembrane-spanning proteins, which included three TRPML proteins (TRPML-1-3, also called MCOLN1-3) [26]. Human TRPML-1 was found to be expressed in several tissues with the highest levels, such as the brain, kidney, spleen, liver, and heart. However, the expression of TRPML-2 and TRPML-3 mRNAs in humans was more restricted [10]. TRPMLs were characterized by their primary intracellular distribution into different subpopulations of membrane vesicles. Besides, TRPMLs were reported to be mainly distributed along the endocytic pathway and participated in the sorting of lipids and proteins [27]. In this study, we firstly investigated the associations between the expression of MCOLN1 and clinical-pathological features of PDAC patients by immunohistochemistry (IHC). 5-year overall survival (OS) and recurrence-free survival (RFS) were analyzed and used to assess the prognosis of patients. A mechanism study confirmed the involvement of MCOLN1 in promoting the PDAC tumor growth both *in intro* and *in vivo*.

Taken together, we provide some significant findings for the target therapy of PDAC.

## 2. Materials and Methods

### 2.1. Patients and Samples

A total of 80 patients pathologically diagnosed with PDAC in Tianjin First Central Hospital were used in our study. The clinical characters of patients such as ages, genders, and pathological features including pTMN stage, tumor grade, tumor size, lymph node metastasis, and vascular invasion were recorded. Tumors were classified according to the 2009 UICC TNM staging as well as in compliance with 2004 WHO/ISUP classifications [18]. This study was approved by the institution ethics commission of Tianjin First Central Hospital, and written informed consent was obtained from participants.

### 2.2. IHC and Scoring

Tumor tissues and matched normal adjacent tissues were fixed into 10% neutral-buffered formalin and were embedded in paraffin. Then, 4 *μ*m sections were cut from paraffin blocks and heated at 65°C for 30 min. Then, tissue sections were performed with EDTA (pH = 8.0) and 3% hydrogen peroxide in methanol. Slides were incubated with a MCOLN1 polyclonal antibody (Cat # OSM00017W, 1 : 500, from rabbit, Invitrogen) at 4°C overnight. Then, the second antibody in the MaxVision™ HRP-Polymer anti-rabbit IHC kit (KIT-5930, Maixin Biology, China) was incubated at room temperature for 30 min, followed by 5 min incubation at room temperature with DAB provided in the kit for color development. The results of MCOLN1 protein expression showed the general cytoplasmic expression. For the results, the proportion of positively stained cells was graded as follows: 0, no positive tumor cells; 1, <5% positive tumor cells; 2, 5-20% positive tumor cells; and 3, >20% positive tumor cells. The intensity of staining was recorded on a scale of 0 (no staining), 1 (weak staining, light yellow), 2 (moderate staining, yellowish brown), and 3 (strong staining, brown). The staining index was calculated as follows: staining index = staining intensity × tumor cell staining grade. High MCOLN1 expression was defined as a staining index score ≥ 4, while low expression was defined as a staining index < 4.

### 2.3. Cell Culture

Two human pancreatic cancer cell lines, PANC-1 and BxPC-3, were obtained from the Cell Bank of the Chinese Academy of Sciences (Shanghai, China). According to the instructions from the American Type Culture Collection (ATCC), PANC-1 cell lines were cultured by RPMI-1640 medium and 10% fetal bovine serum, and BxPC-3 cell lines were maintained in RPMI-1640 supplemented with 10% fetal bovine serum, at 37°C with a humidified atmosphere of 5% CO_2_ in an incubator.

### 2.4. Plasmid Construction and Lentiviral Transfection

MCOLN1 short hairpin RNA oligonucleotide sequence (shRNA) was inserted into the lentiviral vector (Pav-U6-GFP) to construct a MCOLN1-RNAi plasmid. The sequences of shRNA were as follows: 5′-AAGCTGATGCAAGTGGTCAA-3′. The lentiviruses were used to stable transfection. Real-time quantitative PCR and western blot were applied to verify the final effectiveness of knocking down in both cell lines. Qualified cells were selected for later experiments.

### 2.5. Real-Time Quantity PCR

Total mRNA was extracted using the TRIzol (Thermo Fisher Scientific, America) according to the manufacturer's instructions. Then, total RNAs were reverse transcribed to produce cDNA by a cDNA synthesis system, which included 4 *μ*L dNTP-mix, 2 *μ*L primer-mix, 4 *μ*L 5 × PrimeScript buffer, 2 *μ*L DTT, and DEPC water. Quantitative PCR was performed on a Smart Cycler using SGExcel FastSYBR Mixture (with low ROX) Plus (Sango biotech, Shanghai). Forward primers and reverse primers of MCOLN1 were as follows: (F) 5′-TAGCGACTGCCTTCGACCC-3′ and (R) 5′-GCCCTTTTCTCCACCGTGA-3′.

### 2.6. Western Blot

Proteins from different cells were extracted, and the concentration of protein was determined by using the bicinchoninic acid (BCA) method. 50 *μ*g proteins were denatured in sample buffer and then electrophoresed by 10% SDSPAGE. The membranes were blocked and incubated with primary antibodies: rabbit anti-MCOLN1 (1 : 500 dilution, Cambridge, UK), anti-*β*-actin (1 : 1000 dilution, Abcam plc, Cambridge, UK), rabbit anti-Ki67 (1 : 1000 dilution, Abcam plc, Cambridge, UK), and mouse antiproliferating cell nuclear antigen (PCNA) (1 : 500 dilution, Abcam plc, Cambridge, UK) overnight at 4°C. Then, the secondary antibody (polyclonal goat anti-rabbit/mouse, 1 : 10,000 dilution) (Rockland Immunochemicals Inc., Limerick, PA) was incubated for 1 hour.

### 2.7. MTT Array

MTT assay was used to measure the proliferation of PANC-1 and BxPC-3 cells. Cells were seeded into 24-well plates with a density of 2 × 10^3^ cells/well. 10 *μ*L of 5 mg/mL MTT was added into each well and continued to culture for 4 hours. The plates were placed on a microplate autoreader (Bio-Rad, Hercules), and the numbers of cells were measured every day. The assays were performed in triplicate.

### 2.8. Colony Formation Array

300 cells/well of PANC-1 and BxPC-3 cells were seeded into plants for colony formation assay. Finally, the colony formation rate was observed with the naked eye, or under a microscope (low magnification), the colonies in which the number of cells exceeded 50 were counted. The assays were performed in triplicate.

### 2.9. Animal Study

Sixteen athymic Balb/c nude mice, which were born for 5 weeks, were purchased by SLAC Laboratory Animal Co. Ltd. (Shanghai, China). PANC-1 cells transfected with MCOLN1-shRNA and controls were subcutaneously injected into the right armpits of the animals, 2 × 10^6^ cells per animal. The tumor volume was then measured. After inoculation of 29 days, mice were killed and the final tumor tissues were obtained. An animal study was conducted with the approval of the Animal Care and Use Committee of Tianjin First Central Hospital.

### 2.10. Statistical Analysis

SPSS 22.0 software was used for data analysis. According to the variance homogeneity or not, a parametric test and nonparametric test were used, respectively. Associations between the expression of MCOLN1 and the clinicopathological features were evaluated using *χ* ^2^ tests. Associations of survival with MCOLN1 expression were estimated by the Kaplan-Meier method and log-rank tests. Quantitative dates were assessed by mean ± SD, and Student's *t*-test was used in Figures 1 [Fig fig2]–3. For the results, *P* < 0.05 for the difference was significant.

## 3. Results

### 3.1. The Associations between MCOLN1 and Clinical-Pathological Characteristics of Patients with PDAC

To examine the potential link between MCOLN1 and clinical-pathological features of patients with PDAC, a total of 80 PDAC tissue samples obtained from patients after surgery were used to have IHC. The cytoplasm of tumor cells could be dyed, and the typical staining of high and low expression of MCOLN1 is exhibited in Figure 4(a). 80 PDAC tissues (Figure 4(a)) or paracarcinoma tissues (Figure 4(b)) were used to detect the expression levels of MCOLN1 by IHC assays. MCOLN1 in PDAC tissues or paracarcinoma tissues was 51.3% (41/80) and 25.0% (20/80), and the positive rate in PDAC tissues was significantly higher than that that in paracarcinoma tissues (*χ* ^2^ = 11.684, *P* = 0.001 < 0.05). And the results indicated that the expression of MCOLN1 was significantly associated with pTMN stage and vascular invasion. Besides, no obvious associations were found between MCOLN1 expressions with other clinical features, such as age, gender, tumor grade, tumor size, and lymph node metastasis of PDAC patients. The details are summarized in Table 1.

### 3.2. MCOLN1 Was Associated with the Poor Prognosis of PDAC Patients

Then, the Kaplan-Meier method was applied to analyze the association between MCOLN1 expression levels and prognosis. Overall survival (OS) and relapse-free survival (RFS) were followed up. The follow-up in our center was recommended every three months during the first year, then every six months during the following years. Interestingly, data showed that MCOLN1 was obviously associated with OS and RFS. As was shown in Figure 4(b), the high level of MCOLN1 expression was related to the short OS and RFS, suggesting a poor prognosis. In conclusion, MCOLN1 was trending to be an unfavorable factor, which could predict the poor clinical outcomes of PDAC patients.

### 3.3. Lentivirus-Based RNA Interference Effectively Downregulated the Expression of MCOLN1 in Both PANC-1 and BxPC-3 Cells

The expression of MCOLN1 in PANC-1 and BxPC-3 cells was detected by quantitative PCR and western blot. We also stably knocked down the expression of MCOLN1 by lentiviral shRNA constructs each in PANC-1 and BxPC-3 cell lines. As shown in Figure 1, the expression of MCOLN1 in both mRNA and protein levels was dramatically decreased in PDAC cell lines caused by MCOLN1 shRNA transfection. According to these data, we successfully constructed the effective MCOLN1 cell model.

### 3.4. Knocking Down of MCOLN1 Blocked the Proliferation of Cancer Cells In Vitro

The proliferation capacity of PANC-1 and BxPC-3 cells was examined by MTT and colony formation assays. Compared to control, MCOLN1 depletion remarkably inhibited the proliferation of both PANC-1 and BxPC-3 cell lines (Figures 2(a) and 2(b)). To further investigate the roles of MCOLN1 in tumor cell proliferation, the expression of proliferation markers was detected. We found the expression of Ki67 and PCNA was significantly decreased by silencing MCOLN1 (*P* < 0.05, Figures 2(c) and 2(d)). Moreover, we did the test of cell cycle experiment and found that the cells in the G2/M phase were increased while the cells in the S phase were decreased, when the expression of MCOLN1 was depleted in both PANC-1 and BxPC-3 cell lines, respectively (*P* < 0.05, Figure S1). In conclusion, our results revealed that MCOLN1 could promote the proliferation of PDAC cells by regulating the expression of proliferation-relevant proteins including Ki67 and PCNA, and the suppression of MCOLN1 could induce the cell cycle arrest as the G2/M phase.

### 3.5. MCOLN1 Ablation Blocked Tumor Growth In Vivo

To further study the effects of MCOLN1 on tumor growth, PANC-1 cells transfected with MCOLN1-shRNA and control were subcutaneously injected into the right armpits of mice, 2 × 10^6^ cells per animal. Then, tumor volume was measured on the 14th day after injection. Through the growth curve (Figure 3(a)), we found that tumors in MCOLN1 depletion groups were grown slower than control. Besides, the expression of MCOLN1 in two different groups was measured to confirm the effective silencing of MCOLN1 in tumors of mice. The results showed that the expression of MCOLN1 in mRNA and protein levels was reduced caused by MCOLN1 shRNA transfection (Figures 3(b) and 3(c)). Taken together, the results confirmed that MCOLN1 depletion blocked PDAC tumor growth in vivo.

## 4. Discussion

As we know, the mechanism of tumor progression was related to dysregulations of the cell cycle and was accompanied by promoting cell proliferation and/or suppressing apoptosis [19]. The balance between the biological processes of proliferation, apoptosis, and autophagy was regulated by several key factors, such as Ca^2+^, one of the most important regulators of cell survival/death processes [20]. It was found that Ca^2+^ signaling could regulate multiple cellular processes such as cell proliferation, survival, migration, invasion, motility, autophagy, and apoptosis. [21, 22]. As one of the typical Ca^2+^ channels, the TRP channel has been shown to regulate various Ca^2+^-dependent physiological processes in different cell types. [23]. Changes in the activation and/or expression of TRP calcium channels affected calcium-dependent signalling pathways implicated in tumorigenesis and tumor progression [24].

MCOLN1 was a Ca^2+^ channel that releases lysosomal Ca^2+^ and may regulate fusion/fission of vesicles through the endocytic pathway [10–13]. Many studies proposed MCOLN1 as an autophagic regulator, which was necessary for efficient fusion of both autophagosomes and late endosomes with lysosomes [28, 29]. Lysosomal Ca^2+^ release through MCOLN1 could stimulate calcineurin which bound and dephosphorylated its substrate TFEB and thereby promoting its nuclear translocation to initiate autophagy [30]. In addition to MCOLN1, other members of the mucolipin family, TRPML-2 and TRPML-3, were also involved in autophagy regulation [31, 32]. Due to the exact role of MCOLN1 in autophagy, we speculate that it may influence tumor progression through the similar way. Most importantly in the year 2019, the relationship between MCOLN1 and cancer had been studied [14]: MCOLN1 participated in the development of triple-negative breast cancer. Consistent with this result, immunohistochemistry of our study indicated that a high level of MCOLN1 was associated with the poor clinical-pathological features and short survival of patients with PDAC, suggesting that MCOLN1 may play a role in tumor progression of PDAC.

As far as we know, there are a few studies systematically researched on the roles of MCOLN1 in cancer development. Our research was the precedent experiment which systematically studied the role of STK32C in promoting the proliferation in PDAC. Liu et al.'s study found that overexpression of MCOLN1 inhibited imidazole-induced vacuole formation and cell death in human endometrial adenocarcinoma (HEC-1B) cells [16]. In contrast, knockdown MCOLN1 increased the cell death induced by imidazole [16]. Moreover, a report in 2019 demonstrated that MCOLN1 inhibition could attenuate HRAS nanoclustering and plasma membrane abundance, ERK phosphorylation, and cell proliferation [33]. Similarly, in our study, silencing of MCOLN1 obviously inhibits the proliferation of tumor cells. On the mechanism, MCOLN1 depletion inhibited the expression of proliferation cell markers, Ki67 and PCNA. Moreover, suppression of MCOLN1 could induce the cell cycle arrest as the G2/M phase resulting in the inhibition of proliferation. In vivo, MCOLN depletion reduced tumor growth in mice. In summary, our study revealed the link between MCOLN1 and PDAC, which may shed new light on the treatment of PDAC and provide a novel therapeutic target for this cancer. However, the precise molecular mechanisms should be researched and confirmed in the future.

## 5. Conclusion

Our results revealed that the high expression level of MCOLN1 was associated with the poor clinical-pathological characters and predicted the short OS and RFS of patients with PDAC. MCOLN1 inhibited the proliferation of tumor cells in vitro, and silencing of MCOLN1 reduced the tumor growth in mice. In summary, MCOLN1 was a promoting and novel factor in the progression of PDAC.

## Figures and Tables

**Figure 1:** The expression of MCOLN1 in lentivirus-transfected cell lines. The mRNA (a) and (b) protein level expression of MCOLN1 was dramatically decreased in both MCOLN1 shRNA cell lines compared to controls. ^∗^ *P* < 0.05.

**Figure 2 fig2:** The influence of MCOLN1 on the proliferation of PANC-1 and BxPC-3 cell lines by regulating Ki67 and PCNA. (a) The colony formation array showed that the colonies were inhibited in the MCOLN1 shRNA group. (b) The results of MTT showed that the OD value in the MCOLN1 group was lower than that in the control group. (c, d) The expression of Ki67 and PANC was significantly inhibited in the MCOLN1 shRNA group compared to control. ^∗^ *P* < 0.05.

**Figure 3:** In vivo animal experiments. (a) At the 14th day after injection, the tumor volume was measured every day. The growth curve showed that the tumors in the MCOLN1 group grew more slowly than controls. After inoculation of 29 days, the final tumor tissues were obtained. The tumors in the shRNA group were smaller than controls. (b, c) The expression of MCOLN1 in tumors of mice was detected by western blot or IHC. MCOLN1 expression was dramatically decreased in the shRNA group, which confirmed the effective silencing of MCOLN1 in tumors of mice in the shRNA group. “∗” represents the significant association (*P* < 0.05 for the difference was significant).

**Figure 4:** The expression of MCOLN1 in tumor tissues and the associations of MCOLN1 with the prognosis of PDAC patients. (a, b) The staining of high and low expressions of MCOLN1 by IHC in PDAC tissues and paracarcinoma tissues. (c) OS and RFS rates with MCOLN1 expression in the 82 PDAC patients: shorter OS or RFS was significantly observed in high MCOLN1 expression than in low MCOLN1 expression in the 82 PDAC patients (*P* < 0.05, respectively).

**Table 1:** Relationships of MCOLN1 and clinicopathological characteristics in 80 patients with pancreatic ductal adenocarcinoma.

Feature	All *n* = 80	MCOLN1 expression		*χ* ^2^	*P*
		Low	High		
		*n* = 39	*n* = 41		
*Age (year)*				0.450	0.502
<65	64	30	34		
≥65	16	9	7		
*Gender*				0.425	0.514
Male	42	20	24		
Female	34	19	17		
*pTMN stage*				9.881	0.002^∗^
I	22	17	5		
II-III	58	22	36		
*Tumor grade*				0.417	0.518
Low	60	28	32		
High	20	11	9		
*Tumor size*				1.233	0.267
<5	54	24	30		
≥5	26	15	11		
*Lymph node metastasis*				2.818	0.093
Yes	60	26	34		
No	20	13	7		
*Vascular invasion*				4.266	0.039^∗^
Yes	54	22	32		
No	26	17	9		

## Data Availability

The dataset supporting the conclusions of this article is included within the article.

## Supplementary Materials

Supplementary Materials Figure S1: knocking down of MCOLN1 induces cell cycle arrest as G2/M phase.
